# *Leishmania*-Specific Promiscuous Membrane Protein Tubulin Folding Cofactor D Divulges Th_1_/Th_2_ Polarization in the Host via ERK*-*1/2 and p38 MAPK Signaling Cascade

This article has been retracted.

**DOI:** 10.3389/fimmu.2020.00817

**Published:** 2020-06-02

**Authors:** Fauzia Jamal, Manish K. Singh, Jagadish Hansa, Pushpanjali, Ghufran Ahmad, Manas Ranjan Dikhit, Mohd Saad Umar, Sanjiva Bimal, Pradeep Das, Anzar Abdul Mujeeb, Shubhankar K. Singh, Swaleha Zubair, Mohammad Owais

**Affiliations:** ^1^Interdesciplinary Biotechnology Unit, Aligarh Muslim University, Aligarh, India; ^2^Department of Microbiology, Rajendra Memorial Research Institute of Medical Sciences, Patna, India; ^3^Department of Bioinformatics, Rajendra Memorial Research Institute of Medical Sciences, Patna, India; ^4^Department of Immunology, Rajendra Memorial Research Institute of Medical Sciences, Patna, India; ^5^Department of Molecular Biology, Rajendra Memorial Research Institute of Medical Sciences, Patna, India; ^6^Department of Computer Science, Aligarh Muslim University, Aligarh, India

**Keywords:** tubulin folding cofactor D, *Leishmania donovani*, immunoprophylaxis, Th_1_ response, T-cell proliferation, MAPK signaling, peptide cocktail, humoral response

## Abstract

Visceral leishmaniasis (VL)-related mortality and morbidity imposes a great deal of health concern across the globe. The existing anti-leishmanial drug regimen generally fails to eliminate newly emerging resistant isolates of this dreadful parasite. In such circumstances, the development of a prophylactic strategy to impart protection against the disease is likely to take center stage. In order to develop a promising prophylactic vaccine, it is desirable to identify an adequately potential vaccine candidate. *In silico* analysis of *Leishmania* tubulin folding cofactor D protein predicted its potential to activate both B- and T-cell repertoires. Furthermore, the ELISA employing anti-peptide_27_ (a segment of tubulin folding cofactor D) antibody revealed its proficiency in VL diagnosis and treatment monitoring. The peptide_27_ and its cocktail with another *Leishmania* peptide (peptide_23_) prompted the up-regulation of pro-inflammatory cytokines, such as IFN-γ, TNF-α, IL-2, IL-17, *etc*., and the down-regulation of immune-regulatory cytokines, such as IL-10, in the immunized BALB/c mice. Coherent to the consequence of peptide-specific humoral immune response, peptide cocktail-based immunization ensued in the predominant amplification of pathogen-specific IgG2a over the IgG1 isotype, up-regulated proliferation of T lymphocytes, and enhanced production of nitric oxide, reactive oxygen species, *etc*. We also established that the peptide cocktail modulated host MAPK signaling to favor the amplification of Th_1_-dominated immune response in the host. The peptide cocktail mediated the activation of the host immune armory, which was eventually translated into a significant decline in parasitic load in the visceral organs of experimental animals challenged with *Leishmania donovani*.

## Introduction

An uprising trend in the emergence of resistant isolates against available anti-leishmanial drugs has left the healthcare fraternity with limited therapeutic options. Besides the non-availability of effectual drugs, the lack of accurate diagnosis, and treatment monitoring tools is a major obstacle in achieving the effective eradication of visceral leishmaniasis (VL) (1, 2). In the prevailing circumstances, it would be imperative to identify a specific protein-based biomarker that helps in the precise diagnosis of the infection and also acts as a potential antigen to evoke a parasite-specific effector immune response in the host (1, 2). In spite of several ongoing efforts to activate host protective immunity against VL through vaccination, most of the proposed vaccines failed to impart desirable protection. In fact, the development of an effective vaccine against human VL has remained a daunting challenge. The prevalent circumstances warrant the introduction of potent immune-modulators, which can be used along with a candidate antigen to develop a promising vaccination strategy. Our earlier study revealed the presence of numerous potent *Leishmania donovani* antigens in the systemic circulation of infected patients (3). Among several identified parasite antigens, the predominant abundance of tubulin folding cofactor D (TFC-D) along with repertoire of its specific antibodies in circulating immune complexes (CICs) suggests its plausible involvement in the activation of parasite-specific B-cell responses (3).

B-cell epitope mapping has gained significant momentum in recent time and been widely exploited in designing diagnostic, therapeutic, and prophylactic modalities for various biomedical applications (4, 5). In fact, the diversity in size, shape, and structure, and the intrinsic immunogenic attributes of a defensive B-cell epitope can effectively modulate the humoral immune response in the host to fight invading pathogens (5).

Incidentally, a potent subunit vaccine, targeting either *Leishmania* spp. or any other intracellular pathogens, should rather activate effector CD8^+^cytotoxic T lymphocytes (CTLs). In fact, CD8^+^effector CTLs have been evolutionary endowed to eliminate intracellular pathogens as B-cell based humoral immune response has been considered to impart restricted prophylaxis against most of the intracellular pathogens (6). Nevertheless, considerable interest is growing in the vaccinology field to exploit B-cell epitopes in the development of vaccines against many intracellular infections including malaria, salmonellosis, tuberculosis, etc. (7, 8). It has been reported that B-cell can control parasitemia (9) and could be a potential contributor either in designing an effectual vaccine or as an immuno-therapeutic help to clear the VL infection (9–11). Linking T-cell epitopes to a linear B-cell epitope can be considered as a promising vaccine development strategy to improve related prophylactic response in the host (12). It is tempting to speculate that promiscuous epitopes can prime the host immune system and simultaneously boost both T- and B-cell responses in the host. This eventually ensues in the activation of pathogen-specific CD4^+^ Th_1_ cells that have the potential to express cytokines such as interferon-γ (IFN-γ), interleukin-2 (IL-2), interleukine-17 (IL-17), tumor necrosis factor-α (TNF-α), interleukine-12 (IL-12), etc., on one hand and the production of reactive oxygen species (ROS) and inducible nitric oxide synthase (iNOS) on the other. Th_1_ immune response not only primes the host immune defense against primary infection but also imparts life-long immunity against re-infection by the generation of central memory effector cells, a requisite feature for the development of an ideal vaccine candidate (13–15).

In the present study, a holistic approach has been proposed for the simultaneous elicitation of both T- and B-cells along with the mediation of long-term immunity against VL infection (16, 17). The data of the present study establish the vaccine potential of CIC-derived B-cell epitopes and their combination with a potent T-cell epitope to achieve a desirable immune response in the host (3, 14). We also explored the possible involvement of ERK-1/2 and p38 MAPK signaling cascade in the observed host immune cell activation. The study establishes the role of synthetic TFC-D peptide_27_ as a potent diagnostic marker on one hand and its cocktail with another TFC-D fragment, peptide_23_, as an efficient immune-prophylactic prospective vaccine against leishmaniasis.

## Materials and Methods

### Sera Collection

Human serum samples obtained from VL patients were analyzed as per the guidelines of the institutional ethical committee (RMRIMS, Agamkuan, Patna). A total of 124 peripheral blood samples were altogether collected from human subjects (of both sexes in age groups between 18 and 45 years). Sera samples from 25 VL-BT (active VL patients before anti-leishmanial therapy) along with 11 samples each from VL-AT (amphotericin B-treated VL cases: 15 injections of 1 mg/kg weight applied with a very slow infusion of 5% dextrose on alternate days), VL-AT- F (VL patients after 3 and 6 months of follow-up post-treatment), healthy endemic (HE), healthy non-endemic (H-NE), tuberculosis (cases with positive sputum culture), viral (four cases of dengue positive to ELISA, four cases of Japanese encephalitis positive to ELISA, and three cases of influenza A positive to ELISA), malaria (positive to malaria parasite kit), asthma (having chronic airway hyper responsiveness), and filariasis (microfilariae-positive cases of lymphatic filariasis) were procured to perform ELISA (Table S1).

### Computational Elucidation and Cross-Validation of Dominant B-Cell Epitopes

The mass spectrometry (MS) study revealed some potential B-cell epitopes of *L. donovani* (3). We decrypted four abundant epitopes, viz., REAAALLIARL (P_1_), KAEVALFRA (P_2_), ARNELYDMLEIDPPAARA (P_3_), and RAANAGESANE (P_4_), from tubulin folding cofactor D (XP_003861300.1) protein. The third and the fourth epitope sequences (ARNELYDMLEIDPPAARAANAGESANE; named as peptide_27_) were in a linear form with ion score of 42 (ions score >38 indicates identity or extensive homology). The anticipated immunological attributes of peptide_27_ were elucidated by employing a bioinformatics approach. Both the immunogenicity and the physicochemical properties of the targeted epitope were predicted by various immune-informatics algorithms such as Bcepred, ABCpred, and Immune Epitope Database (IEDB) analysis resource. Bioinformatics approaches, viz., Bepipred linear epitope prediction, Karplus and Schulze flexibility, Parker hydrophilicity, Kolaskar and Tongaokar antigenicity, and Emini surface accessibility software, predicted the linear epitope nature, flexibility, hydrophilicity, antigenicity, and surface accessibility of the targeted B-cell epitopes with default thresholds of 0.780, 0.983, 2.4, 0.988, and 1.00, respectively (18–22). The hydrophobicity of the peptide was assessed by *Peptide 2.0* (https://www.peptide2.com/N_peptide_hydrophobicity_hydrophilicity.php) software and *ExPaSy ProtScale* (https://web.expasy.org/protscale/pscale/Hphob.Doolittle.html). The BLASTp (http://blast.ncbi.nlm.nih.gov/Blast.cgi) search was performed against the National Center for Biotechnology Information (NCBI) protein database to retrieve the homolog protein sequences using *L. donovani* XP_003861300.1 as a query. The 1,445-amino-acid sequence of tubulin folding cofactor D with a predicted molecular mass of 154.908 kDa (NCBI accession number: gi|398016223|ref|XP_003861300.1) was retrieved from the Universal Protein Resource database (http://www.uniprot.org/). The primary amino acid sequence was used to search a suitable template in the Protein Data Bank (PDB) to generate 3D coordinates of *Ld* tubulin folding cofactor D. The NCBI BLASTp search did not reveal any suitable template. The tertiary structure was predicted by the Iterative Threading Assembly Refinement (I-TASSER) web server (zhanglab.ccmb.med.umich.edu), which is a hierarchical approach to elucidate protein structure and function. The I-TASSER employs multiple threading approaches (LOMETS) to identify structural templates from PDB. The best five predicted structures were further cross-evaluated by the SAVES server. Based on the C score, the Ramachandran plot, and the ERRAT plot, the best model (model 1) was selected for further analysis.

The conservancy level of the epitope was analyzed by multiple sequence alignment (Constraint-based Multiple Alignment Tool— COBALT, https://www.ncbi.nlm.nih.gov/tools/cobalt/re_cobalt.cgi and Clustal X 2.0) and an epitope conservancy analysis tool from the IEDB analysis resource (http://tools.immuneepitope.org/tools/conservancy/iedb_input). Moreover, to establish the relation with other species, a phylogenetic tree analysis was performed with the BLAST Tree view. The half-life was assessed using ExPaSy ProtParam tool.

### Antigen Detection-Based Serodiagnosis

In order to establish the cross-reactivity of peptide_27_ with the sera of VL-BT and healthy control group, indirect ELISA was performed following the published protocol as standardized in our laboratory (23) (detailed protocol has been included in the Supplementary Methods). The CICs were isolated from peripheral blood and subjected to protein A-mediated antigen dissociation (3). The protein content of the isolated CICs was estimated by employing bicinchoninic acid assay as well as Lowry's method (protein estimation kit; Merck Biosciences). Finally, sandwich ELISA was performed according to the protocol of Sengupta and coworkers (24). The detailed protocol experimental design has been provided in the Supplementary Material's methodology section.

### T-Cell Epitope Analysis

Screening regarding the presence of promising MHC class II epitopes in both peptide_27_ (ARNELYDMLEIDPPAARAANAGESANE) and peptide_23_ (KAEVALFRAHLRRLVTHVTGEDS, _XP_003861300.1_) was executed following the published method (9).

### Mice and Parasites

The present study was approved by the Institutional Animal Ethical Committee of ICMR-RMRIMS, Patna, India. Five- to 8-weeks-old male BALB/c mice, weighing 15–18 g, were procured for this study. A reference strain of *L. donovani* (MHOM/IN/80/Dd8) was cultured and maintained in RPMI-1640 supplemented with 10% fetal bovine serum (FBS) following the published protocol (25). Soluble leishmania antigen (SLA) was prepared following a published protocol and stored at −80°C until further use (26).

### Challenge of Immunized Mice With *L. donovani* Infection

The experimental animals (total 60 BALB/c mice) were divided in the following six groups: (A) unvaccinated mice [immunized with phosphate-buffered saline (PBS)], (B) mice vaccinated with monophosphoryl lipid A (MPLA) and squalene only, (C) mice vaccinated with peptide_27_ plus MPLA/squalene, (D) mice vaccinated with peptide_23_ in combination with MPLA/squalene, (E) mice vaccinated with a cocktail (peptide_27_ + peptide_23_ in 1:1 ratio plus MPLA/squalene), and (F) mice vaccinated with SLA only. Each group consisted of 10 mice. The experiments were repeated at least four to five times to generate statistically significant data. Prior to vaccination, the appropriate dose of antigen to be administered in the experimental animals was determined. To confirm the potency and the immunogenicity of the peptide, the antibody was raised by employing increasing doses (10–30 μg per mouse) of the antigen in mice. The most effective dose (30 μg per animal) was administered in various subsequent experimental setups. The sensitivity of the raised antibody was established with the help of ELISA and Western blotting (Figure S1). The animals belonging to groups C, D, E, and F were subcutaneously immunized with 30 μg each of peptide_27_, peptide_23_, a cocktail of the two peptides, or SLA only, respectively, on days 1, 7, and 15. At 10 days post-administration of the final booster, each group of mice was challenged at dual site intra-cardially and through the tail vein by administering 1 × 10^7^ of freshly transformed *L. donovani* at the early-stationary-phase promastigotes. Three different time points were selected [day 0 post-challenge (PB) and days 30 and 63 post-challenge (PC)] for the assessment of various immunological, biochemical, and pathological parameters. To assess the outcome of the implied immunization protocol, parameters, such as the weight and the size of spleen, anti-leishmanial antibody titer, T-cell proliferation potential (IL-2 and 5-bromo-2'deoxyuridine, BrdU), T-cell function (IFN-γ, TNF-α, IL-10, and IL-17A), downstream signaling pattern (ERK1/2 and MAPK), production of reactive oxygen species and nitric oxide, etc., were ascertained in the immunized mice.

### Induction of IgG1 and IgG2a Response in the Immunized Animals

Humoral immune response was evaluated by measuring the titer of peptide_27_, peptide_23_, cocktail, and SLA-specific mouse IgG1 and IgG2a antibody in the sera of unimmunized and differentially immunized mice by performing indirect enzyme-linked immunosorbent assay (23).

### Preparation of Splenic Mononuclear Cells at Post-Booster and Post-Challenge Stages

Mice from each group, viz., A, B, C, D, E, and F, were sacrificed at various time intervals (PB and PC stage). Spleen was isolated under aseptic conditions and mashed with the help of a frosted glass slide in a sterile dish to obtain a single-cell splenocyte suspension.

### Splenocyte Proliferation Assay

The freshly prepared splenocytes (single-cell suspension) were suspended in RPMI-1640 medium (Sigma, USA) supplemented with 10% fetal calf serum, 2 mM 2-mercaptoethanol (Sigma), and 50 μg/ml gentamycin, 100 U/ml penicillin, and 100 μg/ml streptomycin with pH 7.4. The cells (1 × 10^5^) were plated in 96-well plates and allowed to proliferate for 72 h in a CO_2_ incubator (37°C, 5% CO_2_). BrdU incorporation assay was used to measure the proliferation of splenocytes by employing the BrdU Cell Proliferation ELISA Kit (ab126556).

### Determination of Organ and Gross Body Weight of the Immunized Animals Post-challenge With Infection

The gross body weight of the experimental animals was determined. Next, the spleen size of the representative animal from each group was also determined on day 0 (PB) and PC day 30 and 63 post-challenge stage (PC).

### Determination of Residual Parasite Burden in Splenocytes of *L. donovani* Challenged Mice

The parasite burden was quantified in the splenic tissue smear corresponding to individual mouse from each group at various time intervals. Splenic smear was prepared on glass slides, fixed, stained with Giemsa stain, and manually enumerated under the microscope. The result was recorded as the *Leishmania donovani* unit (LDU), i.e., the number of amastigotes per 1,000 splenocytes per spleen.

### Fluorescence Staining of T-Cells for Qualitative Assessment of Intracellular Cytokines and Mitogen-Activated Protein Kinase Family Proteins

Freshly prepared mononuclear cells (1 × 10^6^ cells/well) from the splenocytes of mice belonging to various immunized groups (at PB and PC stage) were stimulated with various subunit vaccines comprising of synthetic peptide_27_, peptide_23_, peptide cocktail, and SLA control formulation. The cells were incubated in a CO_2_ incubator (5% CO_2_, 37°C) for 24 h. The culture was blocked using Golgi-Plug containing brefeldin A (1 μg/ml, BD) at 4 h prior to harvesting. For the staining of surface markers, the cells were incubated with specific fluorochrome-tagged antibodies, viz., anti-CD3 PE, anti-CD4 PerCP, or anti-CD8 PerCP at 4°C for 20–30 min. After the stipulated incubation, each cell sample was washed with sterile PBS. The cells were fixed by incubating with Cytofix (BD Biosciences) for 30 min at 4°C. The cells were then permeabilized by adding 1 ml perm-wash buffer (1 ×) (BD Biosciences) and further incubated at 4°C for 5 min. Subsequently, the cells were washed and stained with intracellular anti-ERK1/2-PE and anti-p38 MAPK-PE antibody, followed by 30 min of incubation at 4°C. The samples were gently mixed with 1 ml wash buffer (1 ×) and washed thoroughly. The cells were further washed with 2 ml stain solution (PBS with 0.09% NaN_3_ and 1% FBS). Finally, cell pellet was suspended in 500 μl stain buffer and acquired on FACS calibur (BD). The flow cytometry data were further validated using Western blot analysis.

### Quantitative Determination of Various Cytokines in the Immunized Animals by Employing ELISA

Freshly prepared mononuclear cells (1 × 10^6^ cells/well) from the splenocytes of the immunized animals belonging to various experimental groups (on day 0 post-challenge and days 30 and 63 post-challenge) were stimulated with synthetic peptides and incubated in the CO_2_ incubator at 37°C for 72 h. The level of various cytokines, viz., IFN-γ, TNF-α, IL-12, IL-10, and IL-17A, in the culture supernatant was estimated using a commercially available detection kit following the method prescribed in the manuals. Absorbance of the color complex was measured at 450 nm by employing an ELISA reader (Bio-Rad). Variation in the expression level of various cytokines was further validated by reverse transcription polymerase chain reaction (RT-PCR) (method discussed in the Supplementary Materials, methodology section). For this, forward and reverse primers for IFN-γ, IL-12, and IL-10 were designed following the sequence mentioned in Table 1. Likewise, the primer sequence for the TNF-α cytokines was taken from the OriGene website (Rockville, MD, USA).

**Table 1:** List of primers used in semi-quantitative PCR.

**Target gene**	**Product length (bp)**	**Primer sequence**	**Annealing temperature**
Mouse IFN-γ	230	Forward: ATGAACGCTACACACTGCAT Reverse: AGTCTGAGGTAGAAAGAGAT	58
MouseIL-12	220	Forward: TGGAACTACACAAGAACGAGAG Reverse: ACCAGCATGCCCTTGTCTAG	60
Mouse TNF-α	220	Forward: GGTGCCTATGTCTCAGCCTCTT Reverse: CCATAGAACTGATGAGAGGGAG	61
Mouse IL-10	230	Forward: ATGCCTGGCTCAGCACTGCT Reverse: TAACCCTTAAAGTCCTGCAT	56
Mouse GAPDH	220	Forward: TGCATCCTGCACCACCAACT Reverse: TGGGATGACCTTGCCCACAG	60
Mouse iNOS	128	Forward: AGGAGGAGAGAGATCCGATTTAG Reverse: TCAGACTTCCCTGTCTCAGTAG	58

### Measurement of Nitric Oxide and Reactive Oxygen Species

The fresh mononuclear splenocytes (1 × 10^6^ cells/ml/well), isolated from immunized mice belonging to various groups (on day 0 post-challenge and days 30 and 63 post-challenge), were stimulated with antigenic peptides and incubated in the CO_2_ incubator at 37°C for 72 h. Following the stipulated incubation, the level of NO induced in the cultured splenocytes was quantified using a nitric oxide assay kit (Thermo Fisher). The NO concentration was deduced from the standard curve plotted using the known amount of sodium nitrite. Absorbance was measured at a wavelength of 540 nm. The minimum detectable concentration of nitrite was 0.22 mM. Coherently, iNOS concentration was determined by semi-quantitative RT-PCR as well as Western blot analysis by employing anti-iNOS antibody (BD, cat. no. 310329).

For FACS analysis, the freshly isolated splenocytes from the mice belonging to various immunized groups were stimulated with a corresponding antigen preparation at 37°C for 24 h. Next, the cultured splenocytes were washed and further stimulated with 40 μl of n-formylmethionyl-leucyl-phenylalanine (fMLP) (stock of 4 μM FMLP, to get a working concentration of 100 nM for a final volume of 1 ml) at 37°C in a water bath for 10 min. Furthermore, the cell sample was mixed with 50 μl dihydro-rhodamine 123 (DHR) (stock of 200 μM DHR, to obtain a working concentration of 10 μM with a final volume of 1 ml) and incubated at 37°C for 15 min. The sample was treated with 1 ml 1X FACS lysis buffer^TM^ (BD) and centrifuged at 200 × *g* for 5 min. The supernatant was discarded and the pellet was re-suspended in 500 μl of stain buffer (PBS + 1% FBS + 0.09%NaN_3_). The sample was acquired on FACS calibur^TM^ using Cell Quest software (BD). The mean fluorescence intensity corresponding to ROS produced by stimulated cells was measured by flow cytometry.

### Statistical Analysis

Statistical analysis was performed using Graph Pad Prism, version 6.0. The lower limit of positivity (cutoff) of the antigen was established for optimal sensitivity and specificity. The cutoff values (dotted line) for negative and positive sample discrimination were calculated using the mean ± three times the standard deviation of all negative samples. The sensitivity was calculated as the percentage of true positive among the total authentic positive and false negative results. Specificity was calculated as the percentage of true negative and false positive results.

## Results

### Characterization of *Leishmania* Antigens Circulating in the Plasma of VL Patients

Various circulating antigens in the sera of VL patients were characterized using two-dimensional (2D) gel electrophoresis and electron spray ionization liquid chromatography mass spectrometry (ECI-LC-MS). In total, four peptides (P_1_, P_2_, P_3_, and P_4_) were decrypted from a 45-kDa 2D spot analysis. Two sequences in continuity (P_3_ + P_4_) had a high intra-species resemblance (Figure S2A). Moreover, there was no significant similarity of the identified peptides with *Homo sapiens*. The last two 27 mer sequences (P_3_ and P_4_) were fused to get a sequence that was designated as peptide_27_ for further evaluation.

### Computational Elucidation of Dominant Epitopes

The first and foremost aim of the present study was to predict the B-cell antigenic nature of peptide_27_. According to ABCpred, a whole peptide showed an above-the-threshold (0.51) vaccine propensity value. In other words, a bio-informatics study suggested the whole peptide fragment as a potent antigen. Moreover, the BcePred web server predicted all the residues within the peptide sequence ^1^ARNELYDMLEIDPPAARAANAGESANE^27^ as B-cell epitopes, except ^9^LEID^12^ residues. Using various bioinformatics approaches within the IEDB analysis resource, the analysis of Karplus and Schulze demonstrated three discontinuous flexible regions in peptide_27_ (Figure 1A). Furthermore, the Kolaskar and Tongaokar antigenicity prediction tool confirmed the high antigenicity and hydrophilicity of the peptide fragment (^6^NELYDMLEIDPPAARA^18^) with a default threshold (Figure 1B). Moreover, the Parker hydrophilicity prediction established the peptide sequence ^13^PPAARAANAGESANE^27^ as a hydrophilic region. The BepiPred linear epitope prediction revealed ^12^DPPAARAANAGESANE^27^ as a good antigenic region (Figure 1C). Interestingly, the Emini surface accessibility prediction software also displayed most of the residues of the targeted peptide_27_ (^1389^ARNELYDMLEIDPPAARAANAGESANE^1415^) above the threshold value (Figure 1D). Hydrophobicity, determined by Peptide 2.0 software, demonstrated different parameters like hydrophobic 48.15%, acidic 22.22%, basic 7.41%, and neutral 22.22% (Figure 1E). The analyzed data were further validated for the tertiary structure model of tubulin folding cofactor D. In fact, the non-availability of the crystal structure of *Ld* tubulin folding cofactor D prompted us to generate a 3D model (Table 2). The most stable model highlights the epitope region exposed on the surface of the protein (Figure 2). As depicted in Figure 2, most of the amino acid residues occupy the surface region and seem to be highly accessible to the solvent. The surface accessibility assay predicted that the B-cell epitope might be highly accessible to the approaching antibody (27).

**Figure 1:** Computational elucidation of immune dominant epitopes in TFC-D protein employing the immuno-informatics approach. **(A)** Highly flexible amino acid residues (yellow region) present in TFC-D protein. **(B)** The antigenicity of the amino acid residues (6–18th amino acid in the yellow region). **(C)** Linear epitope nature of the amino acid residues involved (^12^DPPAARAANAGESANE${}_{,}^{27}$ yellow region) as revealed by the Bepipred Linear Epitope Prediction software. **(D)** Surface accessibility prediction of whole tubulin folding cofactor D protein. The red circle area represents the peptide sequence (^1389^ARNELYDMLEIDPPAARAANAGESANE^1415^) under study which is above the threshold level. The surface accessibility correlates with the B-cell epitope nature of the targeted peptide sequence. **(E)** The hydrophobicity score of the peptide sequence as predicted by ExPaSy Protscale.

**Table 2:** Stability of the peptide structure of various homology models on the basis of their C score, Ramachandran allowed and disallowed region, Z-score analysis, and Prosa.

**Model**	***C* score**	**Ramachandran allowed and generous allowed region**	**Disallowed region**	**ERRAT**	**PROSA**
1	−1.69	92%	2.6% (33)	86.96%	−9.25
2	−1.98	91.4%	2.7% (35)	80.07	
3	−2.11	89.5%	4.0 (51)	75.61%	
4	−2.36	88.9%	4.1 (52)	74.39	
5	−2.31	87.8%	5.3 (68)	76.40	

**Figure 2:** Computational elucidation for the structural validation of *Leishmania donovani* tubulin folding cofactor D protein. **(A)** C scores of the various homology models prepared in the study as derived by employing the Itasser server. The first model was the best with the least negative C score and low Ramachandran disallowed regions. **(B)** Homology model structure of *L. donovani* tubulin folding cofactor D, with the α-helix, and the β-turn regions shown with different colors (alpha helix, red; beta turn, green; epitope regions, blue). **(C)** Score plot retrieved from ProSA web server represents the model to be within the domicile of the X-ray and the NMR structure. **(D)** ERRAT plot for residue-wise analysis of the best homology model among the five mentioned in Table 2.

Furthermore, MS analysis suggested the peptide_27_ sequence to be conserved among *L. donovani* and *Leishmania infantum* (Figure 3A). Coherently, pBLAST analysis revealed an appreciable percentage identity and a sequence similarity within different *Leishmania* spp. The best 12 BLAST hits had been reported in Figures S2B,C. The sequence had 100% query coverage and 100% identity with *L. infantum*, whereas it had 96% query coverage and 96% identity with *Leishmania major*. The same parameters for *Leishmania braziliensis* and *Leishmania mexicana* were 100 and 85% and 96 and 81%, respectively (Figure S2D). Multiple sequence alignment (MSA) analysis was also conducted through COBALT. Interestingly, an analysis revealed the remarkable sequence similarity between eight *Leishmania* spp., including *L. infantum, L. donovani, L. major, L. braziliensis, Leishmania tarentolae, L. mexicana, Leishmania guyanensis*, and *Leishmania panamensis* (Figure 3A). Blast tree view displayed the phylogenetic relationship with other leishmanial species (Figure 3B). The predicted half-life of the peptide was 4.4 h, which was estimated for mammalian reticulocytes with theoretical pI = 4.08, total number of negatively charged residues = 6, total number of positively charged residue = 2, extinction coefficient = 1,490, Abs 0.1% (or 1 g/L) = 0.516, etc. Moreover, the stability of the peptide was checked *in vivo* by western blot analysis (Figure S1). Non-redundant protein blast did not reveal a significant similarity with other disease-causative agents on one hand and *H. sapiens* on the other. Based on MS data and immuno-informatics evidences, peptide_27_ was selected for further *in vivo* and *in vitro* analysis.

**Figure 3:** Multiple sequence alignment (MSA) and phylogenetic tree. **(A)** An MSA analysis of the TFC-D peptide epitope with other *Leishmania* species suggested a conserved homology within species (analyzed by Constraint-based Multiple Alignment Tool). The area under the box denotes a peptide fragment under study. **(B)** Blast tree view displaying the phylogenetic relationship with other *Leishmania* spp.

### Peptide Synthesis and Its Purity Assessment by Employing HPLC

The peptides were synthesized and assessed for their purity by high-performance liquid chromatography (HPLC). A single peak in HPLC ensured the noise-free peptide synthesis (Figures S3A,B). As mentioned earlier, the purity of the synthesized peptide was also established by 2D gel electrophoresis and ECI-LC-MS. The synthetic peptides were diluted in PBS before their further use in the immunization studies.

### ELISA-Validated Presence of Anti-peptide_27_ Antibody in the Sera of VL Patients

The cross-immune-reactivity of the peptide was assessed by employing sera obtained from various VL-BT and control group patients as revealed by ELISA. The titration curves, as determined by ELISA, suggested that 1 μg of peptide_27_ was appropriate to induce a signal. The frequency distribution graph and the area under the curve (Figures S4A–C) revealed sensitivity of 80% (SeCl; 95%, 69.5–88.5%) and specificity of 100% (SpCl, 86.2–100%) as determined by a software-based statistical analysis that employ the Graph Pad Prism (version 6.0).

### Characterization of Affinity-Purified Anti-peptide_27_ Antibody by Spot ELISA

The specificity of the in-house-prepared rabbit anti-peptide_27_ antibody was established by immunoblotting. The immune-reactivity was confirmed by Western blotting using anti-rabbit secondary antibody (Figure S5A). A band corresponding to 2.8-kDa synthetic peptide_27_ of *L. donovani* was visualized by CBB 250R staining. An affinity-purified anti-peptide_27_-specific antibody exhibited positive reactivity with SLA peptide and negative reactivity with healthy sera, respectively (Figure S5B).

### Determination of *L. donovani* Antigen in CICs Employing Antigen Capture ELISA

An antigen capture ELISA revealed the presence of peptide_27_ in CICs [with optical density (OD) ranging from 0.197 to 0.51] in all the 25 patients with established VL. The OD values for healthy endemic and healthy non-endemic subjects had a range between 0.029 to 0.135 and 0.02 to 0.08, respectively. The OD values for VL-AT and VL-AT-F subjects ranged between 0.042 to 0.175 and 0.025 to 0.125, respectively. However, the OD values corresponding to subjects with viral flu, leprosy, tuberculosis, malaria, and asthma ranged between 0.025 to 0.086, 0.027 to 0.11, 0.031 to 0.23, 0.038 to 0.130, and 0.011 to 0.068, respectively (as shown in Figure 4A). The level of reactivity of CIC with specific antibodies had been depicted by a frequency distribution graph (Figure 4B). The lower limit of positivity (cutoff) was 0.19 for the diagnostic antigen (*P* < 0.0001). Considering VL-BT subject as a test group, with healthy and other disease subjects as the control group, the statistical analysis shows mean ± standard deviation of 0.35 ± 0.07, 0.1 ± 0.04, and 0.02 ± 0.01, respectively (Figure 4C). The area under the receiver operating characteristic curve was 0.994, with a standard error of 0.029, 95% CI of 0.99–1.0, and *P* < 0.0001, respectively (Figure 4D). The ELISA detection revealed the sensitivity to be 96% (SeCl; 95%, 83.28–95.71%) and specificity at 96% (SpCl; 95%, 79.65–99.9 %) as determined by a software-based statistical analysis using Graph Pad Prism (version 6.0).

**Figure 4:** An aliquot of affinity-purified anti-peptide_27_ specific sera (100 μl) at a concentration of 1 μg per well was coated in ELISA plate. The primary antibody was set at a dilution of 1:100. Circulating immune complexes (CICs) present in 1 ml sera sample was used as source of antigen in the sandwich ELISA setup. The horseradish peroxidase-tagged anti-human secondary antibody was used at 1:5,000 dilution. **(A,B)** Frequency distribution of the antigen in visceral leishmaniasis (VL) subjects along with the appropriate control groups. The average of the optical density values for the VL subjects was 5-fold higher as compared to those of healthy controls and other disease subjects. **(C)** Cutoff value at 0.19. **(D)** ELISA revealed 96% sensitivity and specificity with area under receiver operating characteristic curve of 0.994 (*p* < 0.0001). The cutoff values (dotted line) for negative and positive sample discrimination were calculated using the mean ± standard deviation of all the negative samples.

### *In silico* T-Cell Epitope Analysis

Besides B-cell epitope mapping, we also analyzed possible MHC class II-restricted epitopes on the basis of Trost's combining prediction algorithm (28). There was no significant similarity between *L. donovani* TFC-D protein and its *H. sapiens* analog. The 15-mer peptides were predicted to have the binding affinity for the MHC class II-restricted epitope as suggested by SYFPEITHY and IEDB database analysis (Table 3).

**Table 3:** Peptide binding to MHC II molecules of various HLA DRB1 0401-restricted 15 mer epitopes.

**ARNELYDMLEIDPPAARAANAGESANE (Peptide**_****27****_**)**				**KAEVALFRAHLRRLVTHVTGEDS (Peptide**_****23****_**)**			
**IEDB analysis**	Rank*	**SYFPEITHI**	**Score**	**IEDB analysis**	Rank*	**SYFPEITHI**	**Score**
^5^LYDMLEIDPPAARAA^19^	5.99	^5^LYDMLEIDPPAARAA^19^	20	^5^ALFRAHLRRLVTHVT^19^	3.32	^5^ALFRAHLRRLVTHVT^19^	18
^3^NELYDMLEIDPPAAR^17^	5.99	^3^NELYDMLEIDPPAAR^17^	16	^8^RAHLRRLVTHVTGED^22^	4.27	^8^RAHLRRLVTHVTGED^22^	26
^6^YDMLEIDPPAARAAN^20^	6	^6^YDMLEIDPPAARAAN^20^	14	^6^LFRAHLRRLVTHVTG^20^	4.14	^4^VALFRAHLRRLVTHV^18^	22
^4^ELYDMLEIDPPAARA^18^	6.63	^9^LEIDPPAARAANAGE^23^	18	^7^FRAHLRRLVTHVTGE^21^	4.12	^3^EVALFRAHLRRLVTH^17^	20

The MHC class II binding T-cell epitopes analysis was predicted by SYFPEITHY using a matrix-based algorithm and Immune Epitope Database (IEDB, a database which includes the tool that predicts the MHC class I and class II binding epitopes; *Rank, IEBD percentile rank).

### Peptide Cocktail-Based Vaccine Induced Higher IgG2 to IgG1 Ratio in the Immunized Mice

In order to examine the Th1/Th2 cross-regulation and also to decipher the involved protective mechanism, we measured the serum levels of parasite-specific IgG isotypes by employing indirect ELISA (Figures 5A,B). Interestingly, the mice immunized with peptide_27_, peptide_23_, and their cocktail had significantly less abundance of IgG1 antibodies as compared to IgG2a on day 0 (PB) and on days 30 and 63 (PC) post-parasitic challenge (*P* < 0.005). In case of the unimmunized control mice, the level of IgG1 was found to be more elevated as compared to the IgG2a isotype (Figure 5C). The ratio of IgG2a to IgG1 was found to be 2.22, 2.4, and 2.53 in cocktail-vaccinated mice at both PB and PC stages, respectively. The results not only suggest a correlation between humoral immune response and disease control but also establish the role of antibodies in prophylaxis against *L. donovani* infection. The isotype data analysis suggests that the cocktail-based vaccine is a better prophylactic agent as compared to individual peptide_27_- or Peptide_23_-based immune prophylaxis.

**Figure 5:** Determination of IgG1 and IgG2a isotypes in a group of mice differentially immunized with various peptide-based vaccines (*n* = 10) PB (day 0 post-challenge) and PC (days 30 and 63 post-challenge), respectively. **(A)** Absorbance of IgG1 in the sera of animals immunized with various forms of peptide-based vaccines (at 2-fold serial dilutions). **(B)** Absorbance of IgG2a in sera (at 2-fold serial dilutions) of animals immunized with various forms of peptide-based vaccine. **(C)** Heat map showing the ratio of IgG2a to IgG1 in the animal immunized with various forms of vaccines. Data are presented in the form of absorbance mean ± SD. The level of IgG1 and IgG2a isotypes was evaluated using sandwich ELISA. Each experiment was performed thrice and a *P* value <0.05 was considered to be significant.

### T-Cell Activation and Proliferation in Response to Immunization With Novel Subunit Vaccine

The splenocytes isolated from animals immunized with peptide_27_, peptide_23_, and their cocktail showed 3.2-, 1.3-, and 3.6-fold higher T-cell proliferation rate, respectively, as compared to unimmunized mice on day 0 post-challenge (*P* value <0.05). The proliferation increased up to 3.6-, 2.6-, and 4.2-fold and 3.8-, 2.6-, and 4.1-fold in the peptide_27_-, peptide_23_-, and cocktail-immunized groups as compared to the unimmunized control group on days 30 and 63 post-challenge (Figure 6A). The SLA-alone-immunized mice also showed significant T-cell proliferation. However, the magnitude of proliferation was lower as compared to that of the groups of animals immunized with peptide-based vaccines at both PB and PC stages. Improved T-cell activation upon immunization with various peptide-based vaccines was also established by the presence of a significantly higher up-regulation in the expression of IL-2 cytokine. Accordingly, there was at least 1.9-, 3.3-, and 3.7-fold higher production of IL-2 at PB (day 0 post-challenge) and PC (days 30 and 63 post-challenge) as compared to that in the immunized mice. The same trend was observed again in both the cocktail- and the SLA-immunized animals (*P* < 0.005, Figure 6B). Representative dot plots show the gating to a specific T-cell population with CD3^+^ T-cell phenotype and the percentage of CD3^+^ T-cells expressing IL-2 cytokine in various immunized animals (Figure 6C).

**Figure 6:** T-cell activation and proliferation upon immunization with various forms of peptide cocktail-based vaccines. **(A)** Incorporation of 5-bromo-2 deoxyuridine in proliferating splenocytes isolated from various groups of immunized animals at specific time intervals. **(B)** Expression of IL-2 in T-cells isolated from various groups of immunized animals on PB (day 0 post-challenge) and PC (days 30 and 63 post-challenge) as determined by employing FACS Calibur. **(C)** Representative dot plots pertaining to gated CD3^+^ T-cells expressing IL-2. The dot plot data have been shown for the unvaccinated control along with the peptide cocktail-vaccinated mice on days 30 and 63 PC. The bar represents the mean ± SD of four different experiments. Each experiment was performed thrice and a significance *P* value ≤ 0.05 ( ≤ 0.05) was considered to be significant (*p ≤ 0.05, **p ≤ 0.005, ***p ≤ 0.001).

### Immunization With Peptide Cocktail Improves the Efficacy of Vaccine in Terms of the Body Weight and the Spleen Size of the Immunized Mice

In order to establish the efficacy of the in-house-developed peptide_27_-based vaccine as an effective prophylactic candidate against VL, a comparative examination of whole body (Figure 7A) and spleen weight (Figure 7B) with a corresponding change in parasite load in the spleen of mice belonging to various immunized groups was executed (Figure 7C). There was a significant decrease in the parasite load in the spleen of the mice vaccinated with peptides and their cocktail (*P* value <0.005) in comparison to the control groups (unvaccinated and vaccinated with only adjuvant). The maximum parasite clearance was achieved at day 63 (PC). There were 742 amastigotes/1,000 splenocytes and 756 amastigotes/1,000 splenocytes in both control groups of mice on day 63, whereas the mice immunized with peptide_27_, peptide_23_ (individually), or a cocktail of the two peptides had a parasite burden of 92, 116, and 72 amastigotes per 1,000 splenocytes, respectively, at day 63 post challenge (Figure S6). Besides that, mice immunized with SLA also demonstrated efficient parasite clearance (*P* value <0.05). The LDU per spleen was 1.7 × 10^4^ and 7 × 10^5^ at day 30 and 63 in the cocktail-vaccinated mice (Figure 7D). Likewise, SLA also displayed an effective clearance of *L. donovani* parasite.

**Figure 7:** Comparative weight of whole body and spleen as a measure to assess the parasite load in the groups of mice vaccinated with various forms of peptide cocktail. **(A)** Body weight (gram) of mice representing various study groups at different time intervals of day 0 (PB) and days 30 and 63 (PC). **(B)** Spleen weight (in milligrams) at different time intervals in the mice immunized with various peptides at PB and PC stages. **(C)** Representative macrophage ( × 1,000) isolated from various groups of animals showing the *Leishmania donovani* amastigotes (I and II represent the negative and the positive control groups, respectively) (*P* value > 0.001). **(D)** Histogram of the splenic parasitic burden at days 30 and 63 PC in terms of *L. donovani* unit per spleen. Significant values indicate the difference between the immunized and the non-immunized groups (*p ≤ 0.05, **p ≤ 0.005, ***p ≤ 0.001).

### Determination of Cytokine Level by Employing Quantitative ELISA

The quantitative estimation of cytokines was executed by employing sandwich ELISA. The supernatant from cultured splenocytes belonging to various vaccinated mice groups showed a significant variation in cytokine secretion. The expression level of cytokines, viz., IFN-γ, TNF-α, IL-17A, and IL-12, was up-regulated in immunized mice when compared to that of unvaccinated control mice both at PB (day 0 post-challenge) and PC (days 30 and 63 post-challenge) (Figures 8A–D). The expression of IFN-γ was increased by 3.1-, 2.7-, and 3.7-fold in the groups of mice immunized with peptide_27_, peptide_23_, and a cocktail of both, respectively, at day 63 post-challenge (PC 63) (*P* value <0.005) (Figure 8A). Similarly, there was more than 4-fold up-regulation in TNF-α and IL-17A expression level, respectively, in peptide_27_-immunized mice as compared to the unvaccinated controls (*P* value <0.005) (Figures 8B,C). SLA vaccination was also found to boost cytokines in the host; however, the magnitude of the expression was less in comparison to both peptide-alone- as well as peptide-cocktail-immunized groups. The peptide-based immunization induced a low level of IL-10 in the immunized mice (*P* value <0.005) (Figure 8E). The observed cytokine induction pattern suggests a predominant generation of Th_1_-biased response in the host upon immunization with various forms of peptide vaccines_._ Among various peptide-based vaccine candidates, the peptide cocktail-based immunization was most successful in inducing profound pro-inflammatory cytokines in the host. The expression level of various cytokines was further validated by employing reverse transcriptase polymerase chain reaction (Figure 8F).

**Figure 8:** Evaluation of intracellular Th1 and Th2 cytokines expressed by CD4^+^ cells belonging to various groups of animals PB (day 0 post-challenge) and PC (days 30 and 63 post-challenge) (*n* = 10). Quantitative assessment of cytokines, *viz.*, IFN- γ, IL-17, TNF-α, IL-12, and IL-10 as revealed by sandwich ELISA. The representative supernatant from a single-cell suspension of cultured splenocytes belonging to various groups of immunized animals was analyzed for the presence of **(A)** IFN- γ in pg/ml, **(B)** TNF-α in pg/ml, **(C)** IL-17A in pg/ml, **(D)** IL-12 in pg/ml, and **(E)** IL-10 in pg/ml. **(F)** Semi-quantitative PCR for genes specific for IFN-γ, TNF-α, IL-12, IL-10, and GAPDH. Each experiment was performed thrice and a significance *P* value ≤ 0.05 ( ≤ 0.05) was considered to be significant (*p ≤ 0.05, **p ≤ 0.005, ***p ≤ 0.001).

### Peptide Cocktail-Based Vaccination Modulates MAPK Signaling in the Host

In order to assess the potential of various in-house-based peptide vaccines to modulate MAPK family proteins, we determined the expression level of ERK-1/2 and p38-MAPK in the related immune cells. The enzyme p38-MAPK complements the induction of protective signaling in the host. Phosphorylation of ERK1/2 has been correlated with the abundance of anti-inflammatory cytokine IL-10. The pathogens modulate IL-10 expressions to mediate the progression of the disease. The P_27_ peptide alone and its cocktail (with P_23_ peptide) down-regulated the expression of ERK-1/2 in the vaccinated mice in comparison to that of the unimmunized control groups (Figure 9). On the contrary, p38-MAPK was found to be up-regulated in the cocktail-vaccinated mice in comparison to that of the unimmunized control groups (*P* < 0.01). The level of both ERK-1/2 and p38-MAPK was further validated by FACS analysis. The expression pattern of the two MAPK family proteins, namely, ERK-1/2 and MAPK, was further validated by Western blot analysis (Figure 9). All the above specified analyses suggest that the peptide cocktail can down-modulate the expression of ERK-1/2, with a concomitant up-regulation of p38-MAPK.

**Figure 9:** Vaccine-mediated modulation of MAPK signaling cascade as revealed by the estimation of expressed phosphorylated ERK-1/2 and p38 MAPK in CD4^+^ T-cells belonging to various groups of animals immunized with peptide-based vaccines. **(A)** Percentage of CD4^+^ T-cells co-expressing phosphorylated ERK-1/2 in various groups of immunized animals. **(B)** Percentage of CD4^+^ T-cells expressing phosphorylated p38 MAPK in CD4^+^ T-cells belonging to various groups of immunized animals. **(C)** Dot plot showing the mean percentage of CD4^+^ T-cell expressing phosphorylated ERK-1/2 and p38 MAPK on day 30 and 63 in various groups of animals immunized with a peptide-based vaccine. **(D)** Western blot showing the down-regulation of ERK-1/2 and the up-regulation of p38 MAPK in the immune cells of immunized mice. The cell lysate was subjected to SDS-PAGE, followed by blotting to nitrocellulose paper. The blot was probed with specific primary antibodies and horseradish peroxidase-conjugated secondary antibodies at 1:500 and 1:1,000 dilutions, respectively. Each experiment was performed thrice and a value ≤ 0.05 was considered to be significant (*p ≤ 0.05, **p ≤ 0.005, ***p ≤ 0.001).

### Peptide-Based Immunization Boosts Anti-leishmanial Immunity in the Host

Nitric oxide plays a crucial role in the elimination of intra-cellular pathogens, including *Leishmania* amastigotes, during the neutralizing process. We determined the generation of nitric oxide in the splenocytes of differentially immunized animals by employing the Griess reagent. The mononuclear cells isolated from various subunit vaccine-immunized groups of mice showed 3- to 4-fold higher NO expression as compared to that in unvaccinated infected mice on day 63 PC (*P* value <0.005) (Figure 10A). Both western blot analysis and reverse transcription polymerase chain reaction further validated the up-regulated expression of iNOS in the vaccinated mice (Figures 10B,C). Interestingly, the cocktail-vaccinated mice produced the highest levels of NO (*P* value <0.001). SLA-alone vaccination was also successful in up-regulating NO generation; however, the magnitude of expression was significantly less as compared to that of the subunit vaccine-immunized groups.

**Figure 10:** Assessment of leishmanicidal activity in terms of quantitative generation of the nitric oxide (NO) and the reactive oxygen species (ROS) released from macrophages belonging to various groups of immunized animals at PB (day 0 post-challenge) and PC (days 30 and 63 post-challenge). **(A)** Quantitative estimation of NO produced (μM) in the cultured supernatant of the splenocytes. **(B)** Western blot showing the up-regulation of iNOS in vaccinated mice. GAPDH was used as positive control. **(C)** Semi-quantitative PCR for genes specific for iNOS. GAPDH was used as control. **(D)** Reactive oxygen species (ROS) production in the splenocytes. Histogram showing the secretion of ROS by splenocytes isolated from unvaccinated and vaccinated groups of mice PC. The ROS expression data were expressed in terms of mean fluorescent intensity as assessed by flow cytometry. **(E)** Dot plot representative of the oxidative burst of dihydro-rhodamine 123-positive mø. Each experiment was performed thrice and a *P* value ≤ 0.05 was considered to be significant (*p ≤ 0.05, **p ≤ 0.005, ***p ≤ 0.001).

To ascertain whether the peptide-based vaccination translates into parasiticidal activity in the immunized mice, ROS generation was also determined. The splenocytes belonging to peptide_27_-, peptide_23_-, and cocktail-vaccinated mice (at both PB and PC stages) showed a significantly increased oxidative burst in comparison to the unvaccinated or SLA-immunized groups (*P* value <0.005) (Figure 10D). A representative dot plot of the oxidative burst in a DHR-positive cell is shown in Figure 10E. The increased generation of NO and the oxidative burst clearly reflect the potential of peptide_27_-, peptide_23_-, and peptide cocktail-based vaccine in the activation of mononuclear cells to kill *Leishmania* parasite.

## Discussion

In spite of serious global efforts, the development of an effective prophylactic vaccine to eradicate visceral leishmaniasis has remained an elusive task. In the present study, we have tried to establish the immuno-prophylactic potential of an in-house-developed peptide vaccine against experimental visceral leishmaniasis. First, the potent antigen target was identified by employing an extensive immuno-informatics study. The *in silico* analysis suggested the presence of an immunodominant peptide sequence (peptide_27_) in TFC-D, a leishmanial membrane protein which is a primary component of CICs circulating in the bloodstream of VL patients.

The 3D tertiary structure prediction showed the presence of several epitopes on the surface of the TFC-D protein (Figure 2). Appreciating the above-specified facts, we worked on a robust tertiary model of some specific peptides of tubulin folding cofactor D. The model suggested that most of the amino acids of the desired B-cell epitope residues harbor a helical structure (Figure 2B). The presence of helical epitopes, in a given candidate vaccine, is likely to evoke a strong antibody response in the host (20, 21). The surface-exposed epitopes of TFC-D are likely to be recognized by a panel of antibodies (27, 29). The helical conformation is considered to be critical in the recognition of an antigenic sequence (30). It also strongly suggests that the predicted epitope might induce the production of a specific antibody in the host. MSA analysis of the selected peptide assessed the highly conserved region within a species (Figure 3A). The conserved nature of the peptide advocated that it might be used as a target against all the *Leishmania* spp., without any cross-reactivity with humans.

Interestingly, an affinity-purified anti-peptide_27_ antibody exhibited a good cross-reactivity (5-fold more sensitivity) with peptide_27_ and also with the sera of VL patients in comparison to that in the control group. The high level of cross-reactivity establishes the potential of a peptide as an effective biomarker for diagnosis and treatment monitoring. Furthermore, there was no significant similarity found in both TFC-D peptides against any protein of the *H. sapiens* host.

Taking lead from an immune-informatics study, we have tried to explore TFC-D-based small peptides for their immune-prophylactic potential against experimental VL in BALB/c mice. The present work provides an insight to CICs based on TFC-D and their role in the activation of the host immune system (31–33). There are two proline residues in the middle (at 13 and 14 positions) of the peptide_27_ fragment. The proline residues help in the creation of bend and impart flexibility in the epitope region of the peptide. Besides the presence of highly antigenic 6–18th residues, the *in silico* study predicted highly accessible hydrophilic residues in the TFC-D-based peptide_27_. The accessibility as well as the hydrophilicity features is considered to be a desirable attribute of a given B-cell epitope.

Interestingly, the present study also establishes the T-cell epitope attributes of the two peptides derived from TFC-D. In general, Th_1_ response involves the coordinated networking of B, T, and antigen-presenting cell-based cytokines signaling (9, 34). Earlier studies reported the presence of both sero-diagnostic and immune-prophylactic potentials of several *L. donovani* antigens (14, 15). Various fragments of amastigote TFC-D membrane protein seem to have the potential to elicit a desirable immune response in the host. Moreover, the TFC-D based protective B-cell epitopes have also been found to induce the differentiation of *T*_*H*_ cells into effector and memory *T*_*H*_ cells. Such antigenic attributes imply a significant impact on the development of B-cell epitope-based vaccines (35). In fact, both peptides, individually or in a cocktail form, may lead to the development of an efficient vaccine. The proposed peptide cocktail-based vaccine offers a novel target and may help in discovering molecules for best vaccination combinations that direct the differentiation of Th_0_ cells toward the generation of a strong Th_1_ immune response (13). The peptide-based vaccine leads to the generation of central memory T-cells in imparting long-lasting immunity (28).

In the next set of this study, we examined the immunogenicity and the protective efficacy of peptide_27_ against experimental VL in BALB/c mice. Besides being a potent B-cell activator, the *in silico* study suggests the T-cell activation properties of peptides_27_. The immuno-informatics predicted an immune potential of another peptide_23_ that had the potential to substantiate the immunogenicity of linear peptide_27_ in up-regulating the immune response against VL when used as a cocktail of the two peptides (12). The humoral immune response of the peptide cocktail was characterized by evaluating the expression of antigen-specific IgG1 and IgG2a antibody isotype in the sera of differentially immunized mice (Figure 5). The IgG1 antibody expression correlates with an overall Th_2_ response, while IgG2a antibodies are induced in the presence of Th_1_ cell-based cytokines (IFN-γ) (36). The preponderance of IgG2a isotype over IgG1 at both PB and PC stages advocated the better prophylactic efficacy of an in-house-developed peptide-based vaccine against intracellular *L. donovani*.

The immune potential of the cocktail-based vaccine was also evaluated on the basis of the expression level of various signature cytokines by CD4^+^/CD8^+^ cells in the immunized host (37–40). The elevated production of IL-2 also corroborates the expansion of Th_1_ cells in the immunized animals (37). Moreover, the higher expression of other Th_1_ cytokines, namely, IFN-γ and TNF-α, by CD4^+^ cells in the mice vaccinated with the peptide_27_ construct ensured its superior prophylactic potential against infection. The cytokine IFN-γ is a signatory cytokine involved in disease protection, which activates host effector response against parasite-harboring infected macrophages. It may also activate host macrophages to kill parasites through the induction of nitric oxide (41) and reactive oxygen species production (42). The data of the present study explicitly suggest that cocktail-based immunization ensured the higher expression of IFN-γ, TNF-α, and IL-17 in the host (Figure 8). The elevated TNF-α expression in the macrophages might also contribute toward the effective killing of *L. donovani*. (43, 44). The observed killing of the parasite may also find a great correlation with the elevated level of IL-17 cytokine expressed by Th17 cells (45–47). The cytokine IL-17 helps in the protection against VL (46, 47).

On an interesting note, the down-regulation of IL-10 in the immunized mice strongly supports the prophylactic potential of the cocktail-based vaccine against intracellular *L. donovani*. The cytokine IL-10 is a signatory cytokine involved in disease progression, where it blocks Th_1_ activation and consequently down-regulates IFN-γ. It also inhibits macrophage activation for its anti-*Leishmania* activity (48–50). The interaction of master cytokine IL-12 with T-cells helps in the initiation and the maintenance of a Th_1_-type cytokine profile (51) as it regulates the expression of IFN-γ and IL-17. The elevated expression of IL-12 seems to significantly contribute toward an improved outcome of the current peptide-based vaccine.

We observed a significant decrease in *L. donovani* unit in the group of mice immunized with peptide cocktail as compared to that in the unvaccinated control group of mice (Figure 7). The increase in the size and the weight of the spleen belonging to the unimmunized mice can be correlated to parasite burden and the establishment of a full-blown infection. Interestingly, the size of the spleen was normal in the peptide-cocktail-vaccinated mice. The data suggest that the spleen size of the host mouse has a direct correlation with parasite burden.

The generation of the host protective environment has a great correlation with the phosphorylation of various signal transduction-related kinases, including p38 MAPK and ERK-1/2. The ERK-1/2-mediated signal modulation plays a critical role in the survival of the *Leishmania* parasite in the host (52). Intracellular pathogens modulate STAT3/IL-10 praxis and induce alternatively activated macrophages (M2) in the host. The IL-10-mediated anti-inflammatory responses evoke a conducive condition that helps in the survival and the propagation of intracellular pathogens.

The phosphorylation of ERK-1/2 up-regulates IL-10 production, which in turn mediates intracellular parasite proliferation, leading to disease progression. On the other hand, increased phosphorylation of p38 MAPK is associated with an augmented expression of iNOS and IL-12, the two factors that are crucial for parasite eradication (53). The observed enhancement in p38 MAPK phosphorylation with a concomitant decrease of ERK-1/2 phosphorylation in the vaccinated mice suggests the involvement of the two kinases in host protective signaling (Figure 9). The cocktail vaccine revealed better protection for the mice as compared to the peptide_27_-alone treatment_._

The data of the present study establish the potential of *Leishmania* membrane TFC-D peptides to devour the cocktail of a new potent vaccine candidate against human VL. Peptide cocktail-mediated elevated immune response in the host can be attributed to the combined immune activation potential of linear peptide_27_ epitope in conjugation with the overall T-cell repertoire of both peptide_27_ and peptide_23_ (in the cocktail) that led to the simultaneous activation of both B-cells as well as T-cells in the host. The relevance of the peptide_27_-based cocktail needs further validation for its possible wider application as a prospective prophylactic approach against human infection.

## Data Availability Statement

All datasets generated for this study are included in the article/Supplementary Material.

## Ethics Statement

This research was conducted with written informed consent from all subjects in compliance with the recommendations of the Institutional Human Ethics Committee of the Rajendra Memorial Research Institute of Medical Sciences (Patna, India). In accordance with the Helsinki Declaration, all subjects gave written informed consent. The protocol was approved by the Institutional Human Ethical Committee of the Rajendra Memorial Research Institute of Medical Sciences (Patna, India). This research was conducted in accordance with the guidelines of the Animal Ethics Committee of the Rajendra Memorial Research Institute of Medical Sciences (RMRIMS, Patna, India). The protocols were endorsed by the Rajendra Memorial Research Institute of Medical Sciences' (RMRIMS, Patna, India) institutional animal ethical committee.

## Author Contributions

FJ, MO, SZ, and SS conceived and designed the experiments. FJ, MS, P, GA, and MU performed the experiments. FJ, MD, and SZ performed and execute bioinformatics studies. FJ, MD, and AM analyzed the data. PD, SB, SS, SZ, and MO contributed reagents, materials, analysis tools. FJ, SZ, MO, and JH wrote the paper.

## Conflict of Interest

The authors declare that the research was conducted in the absence of any commercial or financial relationships that could be construed as a potential conflict of interest.
